The article "The Efficacy of Rosuvastatin, Amlodipine, and Aspirin in the Treatment of Hypertension with Coronary Heart Disease and Its Effect on Platelet Aggregation" was retracted in 2023. Reasons: unreliable results or conclusions; concerns about the data; concerns about the peer review; concerns about the citations.

# The Efficacy of Rosuvastatin, Amlodipine, and Aspirin in the Treatment of Hypertension with Coronary Heart Disease and Its Effect on Platelet Aggregation

**DOI:** 10.1155/2022/1111438

**Published:** 2022-10-15

**Authors:** Jianli Fu, Ting Wang, Botao Li, Na Zhao

**Affiliations:** Department of Cardiovascular Medicine, Shaanxi Provincial People's Hospital, Xi'an, Shaanxi, China 710068

## Abstract

**Objective:**

This study was to study the efficacy of rosuvastatin, amlodipine, and aspirin in the treatment of hypertension with coronary heart disease and its effect on platelet aggregation.

**Methods:**

The participants included 60 patients with hypertension and coronary heart disease who were treated at our hospital between January 2020 and May 2021 and were randomly assigned to receive either rosuvastatin, amlodipine, and Ziyin Huoxue Recipe (observation group) or rosuvastatin, amlodipine, Ziyin Huoxue Recipe, and aspirin (experimental group), with 30 patients in each. Outcome measures included clinical effectiveness, blood pressure indicators, blood lipid indices, plasma viscosity, platelet aggregation, cardiac function, and adverse responses.

**Results:**

The clinical efficacy in the experimental group was significantly higher than that in the observation group (*P* < 0.05). The differences were found in blood pressure indices and blood lipid indices between the two groups before treatment (*P* > 0.05). However, after treatment, the blood pressure indices in the experimental group were significantly lower than those in the observation group (*P* < 0.05). After treatment, the blood lipid indices, plasma viscosity, and platelet aggregation in the experimental group were significantly lower than those in the observation group (*P* < 0.05). The left ventricular ejection fraction (LVEF) of patients in the experimental group after treatment was significantly higher than that of patients in the observation group (*P* < 0.05). There was no significant difference in the incidence of adverse reactions among patients in the two groups (*P* > 0.05).

**Conclusion:**

The clinical efficacy of rosuvastatin, amlodipine, and aspirin markedly reduces the blood pressure indices, blood lipid indices, plasma viscosity, and platelet aggregation of patients with hypertension and coronary heart disease, improves LVEF, and has a good safety profile.

## 1. Introduction

Hypertension with coronary heart disease is a common cardiovascular disease, with a high prevalence in the elderly [1]. The clinical manifestations include fatigue, palpitations, and angina pectoris. In recent years, the prevalence and mortality of the disease in China have been on the rise [2]. Hypertension and coronary artery disease predispose the patient to disorders of fat and glycemic metabolism and even cause pathological changes in the cardiac and cerebral systems, kidneys, and retina in severe cases. The main pathological manifestation of hypertension is a chronic high blood pressure, often accompanied by dyslipidemia. Lipid abnormalities may promote atherosclerotic lesions in the coronary arteries, leading to adverse cardiovascular events and even death. A close relationship between the risk factors of hypertension and those of coronary heart disease has been reported. Besides, hypertension is an independent risk factor for coronary heart disease. Disease control of hypertension with coronary heart disease is the current clinical challenge [3].

At present, given the absence of specific drugs for hypertension and coronary heart disease, its management is mainly performed empirically. Both hypertension and coronary heart disease damage vascular endothelial cells and increase platelet activity and blood viscosity, which aggravates illness in the coronary arteries [4]. Treatment of patients with hypertension and coronary heart disease mainly focuses on reduction of blood pressure, plasma viscosity, platelet aggregation, and regulation of blood lipid levels. Ziyin Huoxue Recipe is used by our hospital as adjuvant therapy in the treatment of patients with hypertension and coronary heart disease.

Rosuvastatin is a member of statins, which exerts their effects by blocking the HMG-CoA reductase enzyme in the liver. Studies have shown that rosuvastatin plays an important role in the treatment of hypercholesterolemia and hypertension [5]. Amlodipine is one of the dihydropyridine calcium channel antagonists and is commonly used in the treatment of hypertension with a satisfactory clinical effect. It has also been reported that the drug may yield a protective effect on the kidneys [6]. However, Li et al. [7] found elevated platelet activation and blood viscosity in patients with hypertension and coronary heart disease, resulting in increased platelet aggregation and further aggravated disease in the coronary arteries.

Prevention of coronary heart disease is considered essential for the management of hypertensive patients. Aspirin is a nonsteroidal anti-inflammatory drug (NSAID) that is frequently used in the therapeutic setting. NSAIDs block the enzyme cyclooxygenase (COX) to provide analgesic, anti-inflammatory, antiplatelet, and antipyretic effects. Relevant investigations have validated the substantial antiplatelet effect of aspirin, and its involvement in the secondary prevention of coronary artery disease has received much clinical attention. [8]. In traditional Chinese medicine (TCM), coronary heart disease is classified as “true heart pain” and “chest paralysis.” The cause of coronary heart disease is improper diet, internal injury due to fatigue, and internal invasion of cold, with the disease located in the heart. Timely interventions to invigorate blood stasis, activate the meridians, and sedate and calm the mind are necessitated to prevent disease development. The present study is aimed at studying the efficacy of rosuvastatin, amlodipine, and aspirin in the treatment of hypertension with coronary heart disease and its effect on platelet aggregation.

## 2. Material and Method

### 2.1. General Material

60 patients with hypertension and coronary heart disease treated in our hospital from January 2020 to May 2021 were recruited and randomly assigned to either the observation group or the experimental group, with 30 patients in each group. The randomization was carried out using an online web-based randomization tool (freely available at http://www.randomizer.org/). For concealment of allocation, the randomization procedure and assignment were managed by an independent research assistant who was not involved in screening or evaluation of the participants.

#### 2.1.1. Sample Size Estimation

The original sample size calculation estimated that 100 patients in each group would be needed to detect a 3-point difference between groups in a 2-sided significance test with a power of 0.8 and an alpha error level of 0.05.

#### 2.1.2. Ethical Considerations

The study protocol and all amendments were approved by the appropriate ethics committee at each centre. The study was done in accordance with the protocol, its amendments, and standards of Clinical Practice. All participants provided written informed consent before enrolment, Ethics No. HU-TY20200102.

#### 2.1.3. Baseline Information

Of the 30 patients in the observation group, 18 were male and 12 were female. The age of the patients ranged from 42 to 81 years, with an average of 60.58 ± 5.47 years. The duration of disease ranged from 1 to 23 years, with an average of 13.24 ± 4.32 years. Of the 30 patients in the experimental group, 20 were male and 10 were female. The age of the patients ranged from 44 to 80 years, with an average of 60.46 ± 5.39 years. The duration of disease ranged from 2 to 24 years, with an average of 13.22 ± 4.41 years.

### 2.2. Inclusion and Exclusion Criteria

Inclusion criteria are as follows:

1. Patients with a clinical diagnosis of hypertension and coronary heart disease
2. With no contraindications to the use of drugs that were used in this study
3. Who were aware of this study and decided to participate voluntarily
4. With complete clinical data
5. Without other drug treatment
6. Without abnormal liver or kidney function
7. Without malignant tumors
8. Without secondary hypertension or cardiomyopathy
9. Without serious metabolic diseases;
10. Not in pregnancy or lactation

Exclusion criteria are as follows:

1. Patients with serious disease in other organs
2. With abnormalities in coagulation and immune function
3. With mental illnesses or those who were unable to communicate normally
4. Who could not comply or were unable to cooperate with the study

### 2.3. Methods

1. Patients in the two groups were treated with rosuvastatin, amlodipine, and Ziyin Huoxue Recipe. The patients received 10 mg of rosuvastatin (Zhejiang Hisun Pharmaceutical Co. Ltd.; approval number H20143338) daily and 5 mg of amlodipine (Huaishitong Qianlong Pharmaceutical Co. Ltd.; approval number H20103661) daily
2. Patients in the experimental group additionally received aspirin. The patients received 300 mg of aspirin enteric-coated tablets (Bayer Pharmaceutical Health Co. Ltd.; approval number J20080078) daily, and the dose was reduced to 100 mg daily after a month of treatment

## 3. The treatment duration for all patients was 3 consecutive months.

### 3.1. Observational Indicators

1. Treatment efficacy: significantly effective: after treatment, the blood pressure was <140/90 mmHg, the pulse pressure was ≤50 mmHg, with a negative result on double 2-step ladder exercise testing and a normal electrocardiogram (EC G) at rest. Effective: after treatment, there was a decrease in systolic blood pressure (SBP) by less than 30 mmHg, a decrease in diastolic pressure (DBP) by less than 20 mmHg, and a pulse pressure between 50 and 100 mmHg, with a positive result on double 2-step ladder exercise testing and an improvement in the ECG at rest. Ineffective: after treatment, the blood pressure, the pulse pressure, result on double 2-step ladder exercise testing, and the resting ECG met the above stipulated criteria
2. The blood pressure indices (SBP and DBP) of the two groups were measured using a sphygmomanometer
3. Blood lipid indices: the BS-600 automatic blood biochemical analyzer (Shenzhen Mindray) was used to measure the level of total cholesterol (TC) and triacylglycerol (TG) of the two groups of patients
4. Plasma viscosity and platelet aggregation: an automatic blood analyzer was used to measure the plasma viscosity and platelet aggregation in all patients before and after treatment
5. Cardiac function: Doppler ultrasound was used to measure the LVEF in patients before and after treatment
6. Adverse reactions: adverse reactions that may occur during treatment include dizziness, fatigue, nausea, and constipation

### 3.2. Statistical Method

If the parameter beta is either a difference of means, a log odds ratio, or a log hazard ratio, then it is reasonable to assume that *b* is unbiased and normally distributed. SPSS 22.0 software was used as the data analysis software. Measurement data were expressed as $\left(\bar{x}\pm s\right)$ and tested using the independent sample *t*-test. Count data were expressed as the number of cases (%) and analyzed using the *X*^2^ test. Statistical significance was indicated by *P* < 0.05. GraphPad Prism 8 was used to plot the graphics.

## 4. Results

### 4.1. Patient Characteristics

The patient characteristics between the two groups were comparable (*P* > 0.05) (Table 1).

### 4.2. Comparison of Clinical Efficacy

The clinical efficacy in the experimental group was higher than that in the observational group (*P* < 0.05) (Table 2).

### 4.3. Comparison of Blood Pressure Indices

Patients in the observation group had an average SBP of 162.47 ± 12.34 mmHg and 131.86 ± 10.85 mmHg before and after treatment, respectively. Those in the experimental group had an average SBP of 161.87 ± 12.42 mmHg and 114.29 ± 9.64 mmHg before and after treatment, respectively. Patients in the observation group had an average DBP of 103.32 ± 10.35 mmHg and 86.64 ± 10.47 mmHg before and after treatment, respectively. Those in the experimental group had an average DBP of 104.21 ± 10.28 mmHg and 77.59 ± 9.87 mmHg before and after treatment, respectively. The difference in blood pressure indices between patients in the two groups before treatment was not significant (*P* > 0.05). However, after treatment, patients in the experimental group had significantly lower blood pressure indices than those in the observation group (*P* < 0.05) (Figure 1).

### 4.4. Comparison of Blood Lipid Indices

Patients in the observation group had an average TC concentration of 6.33 ± 0.94 and 5.27 ± 0.64 before and after treatment, respectively. Those in the experimental group had an average TC concentration of 6.28 ± 0.89 and 4.36 ± 0.56 before and after treatment, respectively. Patients in the observation group had an average TG concentration of 3.43 ± 0.47 and 2.82 ± 0.36 before and after treatment, respectively. Those in the experimental group had an average TG concentration of 3.45 ± 0.46 and 1.55 ± 0.32 before and after treatment, respectively. Before therapy, there was no significant change in blood lipid indices between the two groups of patients (*P* > 0.05). Patients in the experimental group exhibited considerably lower blood lipid indices following therapy than those in the control group (*P* < 0.05) (Figure 2).

### 4.5. Comparison of Plasma Viscosity, Platelet Aggregation, and LVEF

Patients in the experimental group had reduced plasma viscosity and platelet aggregation after therapy than those in the observational group. The LVEF of the experimental group patients was greater than that of the observational group patients (*P* < 0.05) (Table 3).

### 4.6. Comparison of Adverse Reactions

There was no significant difference in the incidence of adverse reactions between the two groups (*P* > 0.05) (Table 4).

## 5. Discussion

In recent years, the incidence of hypertension has been increasing due to changes in diet and the development of bad habits. Ineffective control of blood pressure will lead to damage of blood vessels and various tissues and organs at all levels. Hypertension with coronary heart disease is one of the most common cardiovascular syndromes in clinical practice. It is considered a major cause of myocardial infarction and heart failure. Modern medicine shows that hypertension is an independent risk factor for the development of coronary heart disease, as it accelerates the progression of coronary atherosclerosis, leading to a rise in ventricular thickness and narrowing of coronary arteries. The hemodynamic changes produced by continuously increasing blood pressure activate platelets in the blood and contribute to atherosclerotic lesions, causing myocardial ischemia, hypoxia, or necrosis, resulting in coronary heart disease. Hypertension results in reduced blood preparation of coronary vessels, causing myocardial hypoxia and ischemia, and the incidence of coronary heart disease is considerably higher in patients with combined hypertension than in those without. Clinical research has gradually evolved from being focused on blood pressure reduction to treatment strategies that are aimed at reducing the comprehensive risk of hypertension [9].

Ma [10] found that because patients with hypertension and coronary heart disease are subjected to the combined effects of both diseases, one-way causality is no longer sufficient to explain and address disease trends and risks. Liang et al. [11] suggested that blood pressure control is not necessarily beneficial in patients with hypertension and coronary heart disease. Patients with coronary heart disease often have increased coronary resistance to blood flow due to long-term atherosclerosis in the coronary arteries. This raises myocardial contractility, which increases intracardiac pressure and coronary artery compression. There is a decrease in coronary blood flow, which, in severe cases, might result in a reversal of coronary blood flow direction. Extremely low blood pressure will lower coronary perfusion pressure and increases the risk of cardiovascular events. Thus, blood pressure regulation in the treatment of individuals with this condition is critical [12].

Amlodipine is a commonly used antihypertensive drug that reduces blood pressure mainly by inhibiting smooth muscle contraction, dilating peripheral blood vessels, and preventing endothelial injury [13]. The medication is frequently used in conjunction with other antihypertensive medications. In TCM, both hypertension and coronary heart disease are linked to the heart, liver, kidneys, and other organs. Because qi deficiency and blood stasis are central to their pathophysiology, the impact of treating several illnesses with the same treatment can be achieved through adequate medication compatibility. Our hospital frequently uses Ziyin Huoxue Recipe as adjuvant therapy in the treatment of patients with hypertension and coronary heart disease. It is a TCM preparation that improves outcome in the management of hypertension and coronary heart disease. Rosuvastatin is one of the commonly prescribed drugs with high treatment efficiency for coronary heart disease [14, 15]. It selectively inhibits the enzyme HMG-CoA reductase to suppress hepatic cholesterol synthesis and reduce the total amount of cholesterol in the blood [16].

Aspirin has remarkable antiplatelet activity and is considered effective in the prevention of thrombosis in patients with coronary heart disease [17].

In the present, the findings revealed that clinical effectiveness in the experimental group was significantly better than that in the control group. This suggests that rosuvastatin, amlodipine, and aspirin outperform rosuvastatin and amlodipine alone, which may be attributed to the strong antiplatelet action of aspirin [18]. In addition, the blood pressure indices and blood lipid indices of the patients in the experimental group after treatment were significantly lower than those of the patients in the observation group. This indicates that rosuvastatin, amlodipine, and aspirin are more effective at reducing blood pressure and blood lipid indices than rosuvastatin and amlodipine alone, which may be ascribed to the lipid-lowering effect by aspirin [18]. Rosuvastatin is a selective HMG-CoA reductase inhibitor that effectively lowers blood lipids and prevents atherosclerosis. It is the best lipid-lowering effect among statins, which reduces intravascular lipid deposition, decreases inflammatory response, delays the formation of atherosclerosis, and inhibits the progression of coronary heart disease. However, its significant modulating effect on cholesterol and LDL cholesterol is considered ineffective for triglycerides and HDL cholesterol, resulting in limited efficacy in the treatment of coronary artery disease [19, 20]. The combination of rosuvastatin, amlodipine, and aspirin may synergistically exert expanded drug properties to potentiate efficacy.

Furthermore, after treatment, the plasma viscosity and platelet aggregation of patients in the experimental group were considerably lower than those of patients in the observation group. It was also discovered that the LVEF of the experimental group after treatment was substantially greater than that of the observation group. This suggests that rosuvastatin, amlodipine, and aspirin are more effective than rosuvastatin and amlodipine alone in lowering plasma viscosity and platelet aggregation. And the results also found that there was no significant difference in the incidence of adverse reactions between the two groups, suggesting a high safety profile of rosuvastatin, amlodipine, and aspirin [14, 21].

The treatment of coronary artery disease complicated with hypertension mainly focuses on vasodilatation to improve blood flow and lower blood pressure. Rosuvastatin calcium tablets reduce lipid deposition and delay the onset of atherosclerosis, amlodipine regulates blood pressure, and aspirin inhibits platelet aggregation, resulting in improved blood flow and reduced blood pressure. However, the cases in the present study were obtained from inpatients in the cardiovascular medicine department of our hospital, which is a single source and a small sample size, and the observation period is short, resulting in limitations in the clinical results. In addition, this study is a clinical study, which provides some references for future treatment and diagnosis. However, this study lacks animal tests to clarify what drug target the combination of these three drugs is based on, suggesting a lack of a more scientific basis. Future studies will further expand the source of cases and sample size, as well as design more indicators and extend the observation period and follow-up, so as to obtain more comprehensive data.

## 6. Conclusion

The clinical efficacy of rosuvastatin, amlodipine, and aspirin markedly reduces the blood pressure indices, blood lipid indices, plasma viscosity, and platelet aggregation of patients with hypertension and coronary heart disease, improves LVEF, has a good safety profile.

## Figures and Tables

**Figure 1:** Comparison of blood pressure indices $\left(\bar{x}\pm s\right)$. NB: ^∗^ denotes *P* > 0.05 and # denotes *P* < 0.05.

**Figure 2:** Comparison of blood lipid indices $\left(\bar{x}\pm s\right)$. NB: ^∗^ denotes *P* > 0.05 and # denotes *P* < 0.05.

**Table 1:** Patient characteristics.

	Observation group (*n* = 30)	Experimental group (*n* = 30)	*t*/*x*^2^	*P*
Sex			0.287	0.592
Male	18	20		
Female	12	10		
Age (years)	42-81	44-80		
Average age (years)	60.58 ± 5.47	60.46 ± 5.39	0.086	0.932
Duration of disease (years)	1-23	2-24		
Average duration of disease (years)	13.24 ± 4.32	13.22 ± 4.41	0.018	0.986

**Table 2:** Comparison of clinical efficacy [*n*(%)].

	Significantly effective	Effective	Ineffective	Total efficacy (%)
Observation group (*n* = 30)	9	14	7	23 (77%)
Experimental group (*n* = 30)	11	18	1	29 (97%)
*x* ^2^	—	—	—	5.192
*P*	—	—	—	0.023

**Table 3:** Comparison of plasma viscosity, platelet aggregation, and LVEF (±s).

	Time	Observation group (*n* = 30)	Experimental group (*n* = 30)	*t*	*P*
Plasma viscosity (mPa·s)	Before treatment	2.12 ± 0.43	2.16 ± 0.41	-0.369	0.713
	After treatment	1.85 ± 0.32	1.33 ± 0.24	7.12	<0.001
Platelet aggregation (%)	Before treatment	88.29 ± 9.42	87.89 ± 10.40	0.156	0.877
	After treatment	75.06 ± 5.63	22.97 ± 6.31	33.738	<0.001
LVEF (%)	Before treatment	37.62 ± 8.34	36.97 ± 9.11	0.288	0.774
	After treatment	41.59 ± 8.42	54.63 ± 6.27	-6.803	<0.001

**Table 4:** Comparison of adverse reactions [*n*(%)].

	Dizziness	Fatigue	Constipation	Nausea	Total incidence (%)
Observation group (*n* = 30)	1	1	0	1	3 (10%)
Experimental group (*n* = 30)	0	2	1	1	4 (13%)
*x* ^2^	—	—	—	—	0.162
*P*	—	—	—	—	0.688

## Data Availability

All data generated or analyzed during this study are included in this published article.
